# Aided Evaluation of Motion Action Based on Attitude Recognition

This article has been retracted.

**DOI:** 10.1155/2022/8388325

**Published:** 2022-03-09

**Authors:** Qi Wang, Qing-Ming Wang

**Affiliations:** ^1^Institute of Mechanical and Dynamic Engineering, East China University of Science and Technology, Shanghai 200237, China; ^2^School of Design and Art, Shanghai Dianji University, Shanghai 200240, China

## Abstract

For athletes who are eager for success, it is difficult to obtain their own movement data due to field equipment, artificial errors, and other factors, which means that they cannot get professional movement guidance and posture correction from sports coaches, which is a disastrous problem. To solve this big problem, combined with the latest research results of deep learning in the field of computer technology, based on the related technology of human posture recognition, this paper uses convolution neural network and video processing technology to create an auxiliary evaluation system of sports movements, which can obtain accurate data and help people interact with each other, so as to help athletes better understand their body posture and movement data. The research results show that: (1) using OpenPose open-source library for pose recognition, joint angle data can be obtained through joint coordinates, and the key points of video human posture can be identified and calculated for easy analysis. (2) The movements of the human body in the video are evaluated. In this way, it is judged whether the action amplitude of the detected target conforms to the standard action data. (3) According to the standard motion database created in this paper, a formal motion auxiliary evaluation system is established; compared with the standard action, the smaller the Euclidean distance is, the more standard it is. The action with an Euclidean distance of 4.79583 is the best action of the tested person. (4) The efficiency of traditional methods is very low, and the correct recognition rate of the method based on BP neural network can be as high as 96.4%; the correct recognition rate of the attitude recognition method based on this paper can be as high as 98.7%, which is 2.3% higher than the previous method. Therefore, the method in this paper has great advantages. The research results of the sports action assistant evaluation system in this paper are good, which effectively solves the difficult problems that plague athletes and can be considered to have achieved certain success; the follow-up system test and operation work need further optimization and research by researchers.

## 1. Introduction

Traditional sports training is faced with some difficult problems, such as venue, equipment, professionals, and difficulty in recording, which are limiting the development of athletes' sports quality. Therefore, designing an auxiliary evaluation system that not only can observe and identify athletes' body posture but also can carry out professional movements according to these athletes' body posture data can help athletes train freely anytime, anywhere, and every moment to the maximum extent and record real and effective real-time records. In this way, the cooperation between sports and computer cutting-edge technology contributes to the intelligence of sports. The article refers to a large number of computer technology journals and sports-related research results, which provides a solid theoretical basis and scientific data support for this article. Video image processing technology is maturing day by day, considering that computer vision involves many fields so far. Various applications (artificial intelligence, pattern recognition, etc.) have a good development trend and are closely related to convolution neural networks in deep learning, so this paper combines several technologies with sports. Reference [1] proposes a rule-based motion recognition algorithm for bone information obtained by depth sensors. Literature [2] designed an aerobics auxiliary evaluation system based on big data and motion recognition algorithm. Literature [3] talks about personal data privacy protection in the era of big data. In reference [4], a new motion recognition method based on key frame and skeleton information is proposed by using Kinect v2 and the weighted K-means algorithm. Reference [5] proposes an improved adaptive human body region segmentation method for human body contour extraction. Reference [6] uses AIC large image data set to understand images more deeply. Reference [7] proposes the FV coding method and automatic scoring technology of human motion features in monocular motion video with local spatio-temporal preservation. Reference [8] proposes a 3D convolution neural network fusing temporal and spatial motion information for human behavior recognition in video. Reference [9] combines optimization algorithm of human posture estimation with deformation model. Reference [10] proposes an acceleration algorithm based on GPU parallel architecture. In reference [11], a point tracking system based on a deep convolution neural network is used to extract feature points and estimate cameras. Document [12] selects machine learning support vector machine algorithm and deep learning framework model for implementation. Reference [13] extracts the descriptor operator of badminton players' motion recognition from video by using the grid classification method of local analysis. Reference [14] proposes a deformable deep scroll neural network for general object detection. Reference [15] proposes a human motion attitude recognition model based on Hu moment invariants and an optimized support vector machine.

## 2. Theoretical Basis

### 2.1. Convolution Neural Network

#### 2.1.1. Overview of Convolution Neural Network

Convolution neural network [16]: *t* description of neurons is shown in Table 1.

“CNN” belongs to a special kind of artificial neuron, as shown in Figure 1.

“CNN” is a favorite of researchers in deep learning methods, and its research results are quite rich and successful in recent years. It is usually used for processes corresponding to natural access and language. Generally, three-dimensional CNN has two operations: convolution and pooling as shown in Figure 2.

The important formulas of the convolution layer are as follows:

(1) $$\begin{array}{c} Z^{l+1}\left(i,j\right)=\left[Z^{l}⊗\omega^{l+1}\right]\left(i,j\right)+b, \end{array}$$

(2) $$\begin{array}{c} Z^{l+1}\left(i,j\right)=\overset{K_{l}}{\underset{k=1}{\sum }}\overset{f}{\underset{x=1}{\sum }}\overset{f}{\underset{y=1}{\sum }}\left[Z_{k}^{l}\left(s_{0}i+x,s_{0}j+y\right)\omega_{k}^{l+1}\left(x,y\right)\right]+b, \end{array}$$

(3) $$\begin{array}{c} L_{l+1}=\frac{L_{l}+2p-f}{s_{0}}+1\;\left(i,j\right)\in \left\{0,1,...L_{l+1}\right\}, \end{array}$$

(4) $$\begin{array}{c} Z^{l+1}=\overset{K_{l}}{\underset{k=1}{\sum }}\overset{L}{\underset{i=1}{\sum }}\overset{L}{\underset{j=1}{\sum }}\left(Z_{i,j,k}^{l}\omega_{k}^{l+1}\right)+b=\omega_{l+1}^{T}Z_{l+1}+b, \end{array}$$

(5) $$\begin{array}{c} L^{l+1}=L. \end{array}$$

The excitation function that assists in expressing complex characteristics, the expression form of Lp pooling, and the linear combination of hybrid pooling are shown in the following formulas:

(6) $$\begin{array}{c} A_{i,j,k}^{l}=f\left(Z_{i,j,k}^{l}\right), \end{array}$$

(7) $$\begin{array}{c} A_{k}^{l}\left(i,j\right)={\left[\overset{f}{\underset{x=1}{\sum }}\overset{f}{\underset{y=1}{\sum }}A_{k}^{l}{\left(s_{0}i+x,s_{0}j+y\right)}^{p}\right]}^{1/p}, \end{array}$$

(8) $$\begin{array}{c} A_{k}^{l}=\lambda L_{1}\left(A_{k}^{l}\right)+L_{\infty }\left(A_{k}^{l}\right),\lambda \in \left[0,1\right]. \end{array}$$

#### 2.1.2. Feature Extraction

In traditional machine learning, the parameters of the classifier can be obtained from the training data, while the feature extractor can be selected. In a convolution neural network, convolution is a feature extractor, and a neural network is equivalent to the classifier. When we train a convolution neural network, it is equivalent to training feature extractor and classifier. We collate some feature extractors designed with convolution neural network, so as to select the most suitable feature extractor for this paper, as shown in Table 2.

The traditional classification model is shown in the following formula:

(9) $$\begin{array}{c} y=f\left(x,\theta classifier\right), \end{array}$$

where *f* represents the feature extraction function, *x* represents the original data, and *θclassifier* represents the classifier.

The expression form of the volume integral class model function is shown in the following formula:

(10) $$\begin{array}{c} y=f\left(x,\theta filter,\theta classifier\right), \end{array}$$

where *θfilter* represents the parameter in the feature extractor.

### 2.2. Human Posture Recognition Technology

Attitude recognition technology finds out the key parts of the human body in images. It is embodied in games, animation modeling, action recognition, and other fields. This technology needs to be optimized all the time to ensure that the recognition of human posture can be very accurate regardless of whether there are clothes shading, the influence of light and shade changes, joints are difficult to observe, and other problems. The site affinity field was selected to treat the key points. In recent years, there are many data sets related to the detection of key parts. Here, as shown in Table 3, we list six commonly used human posture databases.

### 2.3. Action Evaluation Correlation

It is necessary to create and design an action evaluation method suitable for this paper to process the detected human posture data as shown in Table 4.


(11) $$\begin{array}{c} P\left(A|B\right)=P\left(B|A\right)*P\left(A\right)/P\left(B\right). \end{array}$$

### 2.4. Computer Video Processing Technology

#### 2.4.1. Image Correlation Processing

Digital images are represented by two-dimensional arrays.

(1) Grayening of image [23]
  (12) $$\begin{array}{c} Gray=R*0.3+G*0.59+B*0.11, \end{array}$$
  (13) $$\begin{array}{c} Gray=\left(R*30+G*0.59+B*11\right)/100, \end{array}$$
  (14) $$\begin{array}{c} Gray=\left(R*76+G*151+B*28\right)\gg 8, \end{array}$$
  (15) $$\begin{array}{c} Gray=\left(R+G+B\right)/3, \end{array}$$
  (16) $$\begin{array}{c} Gray=G. \end{array}$$
(2) Image binarization
  (17) $$\begin{array}{c} g\left(x,y\right)=\left\{\begin{array}{c} 0\left(Gray\;value\;is\;less\;than\;threshold\left(T\right)\right),\\ 255\left(Gray\;value\;is\;greater\;than\;threshold\left(T\right)\right). \end{array}\right.. \end{array}$$
(3) Enhancement and sharpening
  (18) $$\begin{array}{c} d\left(x,y\right)=f\left(x,y\right)-g\left(x,y\right), \end{array}$$
  (19) $$\begin{array}{c} s_{k}=\overset{k}{\underset{i=0}{\sum }}p_{r}\left(r_{i}\right)=\overset{k}{\underset{i=0}{\sum }}\frac{n_{i}}{n}. \end{array}$$
(4) Edge detection [24]
  (20) $$\begin{array}{c} \nabla^{2}f\left(x,y\right)=\frac{\partial^{2}f\left(x,y\right)}{\partial x^{2}}+\frac{\partial^{2}f\left(x,y\right)}{\partial y^{2}}, \end{array}$$
  (21) $$\begin{array}{c} \nabla^{2}f\left(x,y\right)=f\left(x+1,y\right)+f\left(x-1,y\right)+f\left(x,y+1\right)+f\left(x,y-1\right)-4f\left(x+1,y\right). \end{array}$$

#### 2.4.2. Motion Video Correlation Processing

(1) Video Transform [25]
The video camera finally outputs the RGB format video image. Converting it to HSV format can reduce the image preprocessing time and improve the overall efficiency of image recognition after image processing, as shown in Figures 3 and 4.
The relevant formula is expressed as follows:
  (22) $$\begin{array}{c} H=\left\{\begin{array}{c} 0,\max=\min\\ 60\times \frac{G-B}{\max-\min}+0,\max=r,G\geq B\\ 60\times \frac{G-B}{\max-\min}+360,\max=r,G<B\\ 60\times \frac{B-R}{\max-\min}+120,\max=G\\ 60\times \frac{R-G}{\max-\min}+0,\max=B \end{array}\right., \end{array}$$
  (23) $$\begin{array}{c} S=\left\{\begin{array}{c} 0,\max=0\\ 1-\frac{\min}{\max},\max\neq 0 \end{array}\right., \end{array}$$
  (24) $$\begin{array}{c} V=\frac{\max}{255}. \end{array}$$
(2) Compensation of motion residuals
 When the human body moves, it is easily interfered by light and shadow or external signal environment, including color shift, loss, jitter, abnormal brightness, and so on. At this time, motion residuals will appear. When calculating the residual value of each pixel, we can set the energy law index of the video image together. The formula for calculating the residual value is as follows:
  (25) $$\begin{array}{c} \left\{\begin{array}{c} \Delta_{loss}\left(x,y\right)=f\left(x,y\right)\left[1-P\left(x,y\right)\right]\\ \Delta_{weighted}\left(x,y\right)=f\left(x,y\right)P\left(x,y\right)\\ \Delta_{pres}\left(x,y\right)=\Delta_{loss}\left(x,y\right){\left[1-SA\left(x,y\right)\right]}^{\rho }\\ f\left(x,y\right)=\Delta_{weighted}\left(x,y\right)+\Delta_{pres}\left(x,y\right) \end{array}\right., \end{array}$$
 where Δ_*loss*_(*x*, *y*), Δ_*weighted*_(*x*, *y*), and Δ_*pres*_(*x*, *y*) represent the weighted residuals perceived by video images; *P*(*x*, *y*) and *SA*(*x*, *y*), respectively, representing the residual value of each pixel and the space in the video scene; and *ρ* represents the exponent of the set energy law.
(3) Image filtering
  (26) $$\begin{array}{c} I_{mid}=Med\left\{i\right\}=\left\{\begin{array}{c} I_{i\left(\frac{n+1}{2}\right)},n\;is\;an\;odd\;number\\ \frac{1}{2}\left[I_{i\left(\frac{n}{2}\right)}+I_{i\left(\frac{n+1}{2}\right)}\right],n\;is\;an\;even\;number \end{array}\right., \end{array}$$
  (27) $$\begin{array}{c} g\left(x,y\right)=Med\left\{f\left(i,j\right),\left(i,j\right)\right\}. \end{array}$$
(4) Similarity between feature vectors of human motion posture
  (28) $$\begin{array}{c} Sim\left(i,j\right)=\left|BR\left(i\right)-BR\left(j\right)\right|. \end{array}$$

## 3. Motion-Aided Evaluation System Based on Attitude Recognition

### 3.1. Moving Target Detection

The most important step in the system is to process the computer video when carrying out the auxiliary evaluation of sports actions. Only when the moving target is detected smoothly can the following series of operation processes be realized, as shown in Figure 5.

Firstly, we construct the background model of the video image. Its principle is that the capture time interval of each frame of moving image is short, and several frames of images recorded by us are at the same position, so the position is the background pixel. And pixel combinations can get accurate background images. The pixel value and gray value of the background image are unified, and the background is subtracted to obtain the moving area of the target. Whether the pixel value changes in the area is observed in several consecutive video frames, so as to determine whether the target in the area is in a moving state.

### 3.2. Human Posture Recognition Module

#### 3.2.1. OpenPose Attitude Recognition

We chose the OpenPose open-source library, and the training set is provided by CMU Panoptic Studio. This algorithm can detect real-time, multitarget selection, in the recognition of the human body in many of the research obtained a lot of successful cases, so there are many cases that can be referred to. The affinity field is used to associate key body parts. It can effectively detect the 2D action posture of a single person or multiple people in the video image to be detected. Finally, the coordinate file with body key points marked on the detected target on the original image is output.

(29) $$\begin{array}{c} L^{t}=\phi \left(F,L^{t-1}\right),\forall 2\leq t\leq T_{p}, \end{array}$$

(30) $$\begin{array}{c} S^{T_{P}}=\rho^{t}\left(F,L^{T_{P}}\right),\forall t=T_{P}, \end{array}$$

(31) $$\begin{array}{c} S^{t}=\rho^{t}\left(F,L^{T_{P}},S^{t-1}\right),\forall T_{P}<t\leq T_{P}+T_{C}. \end{array}$$

The key points obtained by this module should be accurate and conform to the normal motion posture extraction, so as to evaluate correctly, as shown in Figure 6.

#### 3.2.2. Application of Motion Evaluation Method

As shown in Figure 7, the premise of action recognition also needs to deal with things describing action rules. When we describe the action, we can use the joint points of the human body to calculate the joint angle of the human body by finding a cosine angle with known three-point coordinates. Eight joint angles were selected as human movement indexes, as shown in Table 5.

### 3.3. Design and Implementation of the System

#### 3.3.1. System Development Platform

It is shown in Table 6.

#### 3.3.2. Overall Design of the System

*The General Design of Motion Attitude Recognition Process.* As shown in Figure 8, two databases are created during the recognition of motion posture. These two databases are very important, one of which can capture human motion; the other is a database of processed human motion characteristics. Every step is fully considered in the whole process design, whether it is the interception and capture of video images or the feature matching of data and so on. Through our process, we can give more accurate recognition results in detail.

*Design of the Aided Evaluation System for Motion.* As shown in Figure 9, before logging in, you must register your identity to ensure security and privacy. During the whole operation process, the system will automatically save all the data every 5 min with the increase of time and store them in the information center of the user. If the user stops using it, the system will immediately save all the test-related information. After more than 20 min, the system automatically shuts down. After the system is shut down, if the user needs to use it, he must reopen the interface, open his own data repository, and reopen the interface.

*The Personal Information Module Has Special Password Management.* Standard action database provides the most powerful support for the database system, and the application of data needs this module to participate. Here, it will open the picture to be processed for posture feature extraction and find the joint angle of the detected target as an evaluation reference. Of course, this part will also provide the function of adding actions and deleting actions.

As its name implies, the auxiliary teaching module provides users with an opportunity to practice. After getting the joint angle, users can compare the similarity between the actions in the database and the actions in the database and, finally, output the final detection results.

All the functions of the overall evaluation module are offline, and users can use the functions without hindrance without a network.

## 4. Experimental Analysis

### 4.1. OpenPose Attitude Recognition Effect

The configuration environment is shown in Table 7.

The key nodes of the human skeleton model are identified as shown in Figure 10.

As shown in Figure 11, we invited a volunteer participant as our pretester.

The joint point coordinate data are collated as shown in Figure 12. The joint coordinates are obtained to calculate the joint angle. By getting the joint angle, we can accurately determine the key points of our human posture. Because the participant's right foot is blocked, the joint coordinates of the action are missing “right foot,” which is the shortcoming of the system designed in this paper.

### 4.2. Action Evaluation Pretest

We invited three volunteers to pretest the same action, as shown in Figure 13.

The comparison is shown in Figure 14.

Everyone's force point and posture are different. Although all three participants made the action of lifting dumbbells horizontally, the women's hands in the middle picture are basically parallel to the ground, and the two men's arms in the left and right pictures are inclined to the ground in different degrees, but their postures are generally the same. According to the joint angle number corresponding to the joint in Table 5, we can know whether their motion amplitude meets the standard data.

### 4.3. Test of Sports Action Auxiliary Evaluation System

#### 4.3.1. Overall Evaluation of the System

The overall system interface is shown in Figure 15.

The basic toolbar has basic functions, such as file import and export, editing class operations, view selection, and seeking help. The function module is mainly to realize the core functions of the main design of the four systems. The center of the system interface is a large area, which is mainly the video image processing area. We can intuitively observe the whole process. Below this area, there are four functions for processing: action selection, start detection, pause processing, and stop processing. The rightmost column is about the horizontal and vertical coordinates of the key points of the human body detected and processed by us and the corresponding current confidence level.

A database is established (i.e., the standard action database mentioned above), and we collect up to 200 motion video sequences (evenly distributed into 15 categories) for auxiliary comparison reference of motion actions. As shown in Figure 16, we (partially) intercepted the joint angle data of 5 standard movements in the database for display.

If two different people are doing the same action, if you want to know who is doing it more standard, you need to use a method to find the “distance” between the two actions: minimum Euclidean distance, that is, the similarity measure between two actions. The formula related to Euclidean distance is as follows:

(32) $$\begin{array}{c} d\left(x,y\right)={\left(\overset{n}{\underset{i=1}{\sum }}{\left(x_{i}-y_{i}\right)}^{2}\right)}^{1/2}. \end{array}$$

As shown in Figure 17, we invited a volunteer participant to record the video. We select a video action frame similar to standard actions 1 and 2 for joint angle data display. We can know that the number of action frames A most similar to standard action 1 is 4, and the Euclidean distance from standard action 1 is 5.09902; the number of action frames B most similar to standard action 2 is 7, and the Euclidean distance from standard action 2 is 4.79583. The best action of this participant is the action with the smallest Euclidean distance, that is, the action with Euclidean distance of 4.79583.

If the participant wants to perfect and standardize his movements, he needs to use the auxiliary teaching function given by this system to practice frequently, approach the standard joint angle data as much as possible, and reduce the Euclidean distance between his movements and the standard movements.

#### 4.3.2. Experimental Result Data

We conducted an action-assisted evaluation on seven kinds of sports videos. The video is set up as shown in Table 8.

Of course, in order to better explain the superiority of our system experimental results, we choose to make a comparison with the recognition method based on BP neural network and the traditional recognition method, as shown in Figure 18.

We can see from Figure 18 that the traditional method is extremely inefficient, in which the error rate of sit-ups can be as high as 6.8%, and the recognized results are too different from the real results. The recognition method based on BP neural network has obviously improved, and its correct recognition rate can be as high as 96.4%, which is very close to the real result. The correct recognition rate of this method can be as high as 98.7%, which is 2.3% higher than that of the recognition method based on BP neural network. Therefore, this method is the most superior recognition method, and there is room for further optimization in the follow-up work.

## 5. Conclusion

This paper combines computer technology with sports direction, obtains very ideal data results, verifies the feasibility of this system, makes sports glow with new vitality, and takes a big step forward to intelligence.

The results show that

1. The joint angle data can be obtained from joint coordinates, and the key points of human posture can be calculated for easy analysis.
2. Motion evaluation criteria is used to measure the video human posture, so as to judge the detection.
3. According to the standard motion database created in this paper, a formal motion auxiliary evaluation system is established; compared with the standard action, the smaller the Euclidean distance is, the more standard it is. The action with an Euclidean distance of 4.79583 is the best action of the tested person.
4. Efficiency and inefficiency of traditional methods: the correct recognition rate based on BP neural network method is 96.4%. The correct recognition rate of the attitude recognition method based on this paper can be as high as 98.7%, which is 2.3% higher than the previous method; therefore, the method in this paper has great advantages and the system research results are satisfactory.

In this paper, due to technical limitations, we need to further study the fine optimization. It is still in the initial stage, and a large number of deep problems need to be studied. In the recognition process, the problems such as small target, ambiguity, and occlusion will affect the final result, so the automatic recognition rate of attitude motion can further expand the rising space.

## Figures and Tables

**Figure 1:** Artificial neuron.

**Figure 2:** Single-layer convolution neural network.

**Figure 3:** RGB color space representation.

**Figure 4:** HSV color space representation.

**Figure 5:** Flow chart of moving target detection.

**Figure 6:** Workflow of human posture recognition module.

**Figure 7:** Action description rule workflow.

**Figure 8:** Flow chart of automatic motion attitude recognition.

**Figure 9:** Overall function of the system.

**Figure 10:** Human skeleton model diagram.

**Figure 11:** Joint point coordinates.

**Figure 12:** Joint point coordinates.

**Figure 13:** The same action model diagram of three participants.

**Figure 14:** Comparison of joint angle data of three participants.

**Figure 15:** System interface.

**Figure 16:** (Standard) joint angle data.

**Figure 17:** Joint angle data similar to standard actions 1 and 2.

**Figure 18:** Experimental comparison results of correct identification quantity.

**Table 1:** Description of neurons.

A natural neuron	
Composition	Neuronal nucleus
	Dendrites [17]
	Axon

Explanation: Axons are branched off to connect with dendrites of other neurons to form synapses. Artificial neurons have a similar structure, which also contains a nucleus (processing unit), multiple dendrites (similar to the input), and an axon (similar to the output).	

**Table 2:** Feature extractor based on convolution neural network design.

Name	Description
LeNet [18]	Proposed by LeCun in 1998, it is the first CNN. It has a seven-level convolution network dedicated to classifying numbers and has the ability to classify numbers without being affected by minor distortion, rotation, and changes in position and scale.

AlexNet	Proposed by Krizhevesky et al., by deepening CNN and applying many parameter optimization strategies to enhance CNN's learning ability, it is considered as the first deep CNN architecture, showing the pioneering achievements of image classification and recognition tasks.

ZefNet	It is recognized as the winner of ILSVRC (CNN competition) in 2013. It uses deconvolution to visually analyze CNN's intermediate feature map, finds a way to improve the model by analyzing feature behavior, and fine-tunes AlexNet to improve its performance. It manages to achieve a Top-5 error rate of only 14.8%. This achievement of ZefNet is achieved by adjusting AlexNet's super parameters and keeping the same structure. In order to further improve the effectiveness and accuracy of ZefNet, more deep learning elements have been added.

GoogleNet	GoogleNet, which won the 2014-ILSVRC competition, introduced a new concept of inception blocks into CNN, integrating multiscale convolution transformations through split, transform, and merge ideas. This block encapsulates filters of different sizes (1 × 1, 3 × 3, and 5 × 5) to capture spatial information of different scales (fine-grained and coarse-grained). In addition to improving learning ability, GoogleNet focuses on improving the efficiency of CNN parameters.

VGG [19]	With the successful application of CNN in image recognition, Simonyan et al. put forward a simple and effective design principle of CNN architecture. Their architecture, called VGG, is a modular layered pattern. VGG has a depth of 19 layers to simulate the relationship between depth and network presentation ability. VGG replaces 11 × 11 and 5 × 5 filters with a stack of 3 × 3 convolution layers. Experiments show that placing 3 × 3 filters at the same time can achieve the effect of large-size filters.

**Table 3:** Examples of 2D human posture data set.

Data set	Type	Number of joint points	Number of samples/103	Usage
LSP	Single person	14	2	Basic abandonment
FLIC	Single person	9	20	Basic abandonment
MPII [20]	Single person, multiple person	16	25	Mainstream
MSC0C0	Multiple persons	17	>300	Mainstream
AI challenger	Multiple persons	14	380	Competition only
PoseTrack [21]	Multiple persons	15	>20 frame	Most of them are used for attitude tracking

**Table 4:** Motion evaluation method.

Method	Description
Template-based method	In the matching mode, the action sequence to be detected is compared with the pre-established style action library according to a specific time order, and the action similarity is introduced to evaluate the action. When encountering complex action, we don't need to pay attention to the time order when studying its action. We can use the dynamic matching method to compare and analyze the actions at any time in the action sequence to be detected with the style action library. Next, find the best way to match these two methods to achieve the effect of motion recognition and classification.

Method based on state space [22]	The hidden Markov (HMN) model is one of the most convincing methods in this type of action evaluation. Researchers put forward Bayesian network based on probability inference, which eliminates uncertainty and incompleteness. Compared with the link structure of HMN, Bayesian network is a directed graph describing a random process, which well expresses the time and sequence transformation of the state.

**Table 5:** Selection of joint angle.

Joint angle number	Joint point
1	Head, neck, left shoulder
2	Left shoulder, left elbow, left wrist
3	Right shoulder, right elbow, right wrist
4	Left elbow, left shoulder, left hip
5	Right elbow, right shoulder, right hip
6	Left knee, neck, right knee
7	Left hip, left knee, left foot
8	Right hip, right knee, right foot

**Table 6:** Main configuration.

Hardware platform	Software platform
CPU: Intel (R) core (TM) i5-8300H 2.30 GHz; GPU: NVIDIA GeForce GTX1050Ti 4G; disk: Samsung MZVLB256HAHQ 237G; memory: Samsung DDR4 2666 MHz 8 GB	The software platform is mainly built in visual studio 2015 environment. Open-source computer vision library OpenCV, Microsoft MFC interface library, CUDA architecture, and GPU acceleration library cuDNN are used. The system uses C++ for development, using C++ file operation classes of stream, if stream involved in the program files, data types, text flow, and other objects for processing.

**Table 7:** OpenPose configuration environment.

Type		Parameter
Hardware environment	Operating system	Windows 10 Home Edition
	CPU	Intel® core I5–8300H
	Graphics card	Nvidia GTX1050Ti
	Memory	Samsung 8 GB

Software environment	Integrated development environment	Visual studio 2015, cmake
	Acceleration library	CUDA 8.0, CUDNN 5.5

**Table 8:** Experimental test video settings.

Video name	Format	Frame number	Storage space (MB)
Walk	1,280 × 720	300	644
Swimming	1,280 × 720	900	592
Running	1,920 × 1,080	600	411
Sit-ups	1,920 × 1,080	504	508
Pull-up	1,280 × 720	600	555
Basketball	1,920 × 1,080	600	623
Skipping rope	1,920 × 1,080	500	517

## Data Availability

The experimental data used to support the findings of this study are available from the corresponding author upon request.
